RETRACTED

# Tbx1 Regulates the BMP-Smad1 Pathway in a Transcription Independent Manner

**DOI:** 10.1371/journal.pone.0006049

**Published:** 2009-06-25

**Authors:** F. Gabriella Fulcoli, Tuong Huynh, Peter J. Scambler, Antonio Baldini

**Affiliations:** 1 Telethon Institute of Genetics and Medicine, Naples, Italy; 2 Institute of Biosciences and Technology, Texas A&M University Health Sciences Center, Houston, Texas, United States of America; 3 Institute of Child Health, London, United Kingdom; 4 University Federico II, Naples, Italy; 5 Institute of Genetics and Biophysics, CNR, Naples, Italy; The University of Hong Kong, China

## Abstract

Tbx1 is a T-box transcription factor implicated in DiGeorge syndrome. The molecular function of Tbx1 is unclear although it can transactivate reporters with T-box binding elements. We discovered that Tbx1 binds Smad1 and suppresses the Bmp4/Smad1 signaling. Tbx1 interferes with Smad1 to Smad4 binding, and a mutation of Tbx1 that abolishes transactivation, does not affect Smad1 binding nor does affect the ability to suppress Smad1 activity. In addition, a disease-associated mutation of TBX1 that does not prevent transactivation, prevents the TBX1-SMAD1 interaction. Expression of *Tbx1* in transgenic mice generates phenotypes similar to those associated with loss of a Bmp receptor. One phenotype could be rescued by transgenic *Smad1* expression. Our data indicate that Tbx1 interferes with Bmp/Smad1 signaling and provide strong evidence that a T-box transcription factor has functions unrelated to transactivation.

## Introduction

Tbx1 is a T-box transcription factor required for pharyngeal and cardiovascular development of humans and mice [1]–[3]. Mutations in *TBX1* cause DiGeorge syndrome [4]–[6] and its molecular functions are unknown, but it can transactivate reporters with T-box binding elements [6]–[8]. T-box proteins, including those of the Tbx1 subfamily may interact with histone modifying enzymes H3K27-demethylase and H3K4-methyltransferase and thus modulate gene expression [9]. We and others have identified a number of genes potentially targeted by Tbx1 [7], [10]–[13], but the mechanism(s) by which it can regulate the transcription of these genes and how it controls developmental pathways is unclear. A major obstacle to understanding these mechanisms is our poor knowledge of the molecular interactors of Tbx1. One of the best studied developmental functions of *Tbx1* is in heart development, where it is required to sustain proliferation of mesodermally-derived cardiac progenitors of the second heart field (SHF), a cardiac progenitor cell population that contributes to the development of most of the heart, including the outflow tract and right ventricle [7], [14]. Recent data have shown that loss of function of *Tbx1* is associated with increased expression of differentiation markers of the myocardium, suggesting that *Tbx1* may also regulate negatively cardiomyocyte differentiation [13]. The mechanisms and gene networks that regulate the homeostasis of the SHF cell population are not completely understood. However, it is clear that major signaling systems, such as the fibroblast growth factor (FGF) and bone morphogenetic protein (BMP), as well as transcription factors such Nkx2.5, Isl1, Tbx1 and Foxh1 contribute to specification, proliferation and/or maintenance of this population [15]. In particular, it has been shown that Nkx2.5 regulates negatively the expression of Bmp2, establishing an Nkx2.5/Bmp2/Smad1 negative feedback loop that regulates proliferation of cardiac progenitors of the SHF [16]. Here we show that Tbx1 contributes to this network in an unexpected manner, i.e. by binding to Smad1, interfering with Smad1-Smad4 dimerization and suppressing its transactivation ability.

RETRACTED

## Results

### Tbx1 binds Smad1

To identify Tbx1 interacting proteins in mammalian cells, we performed affinity purification of Tbx1-interactors complexes followed by identification of co-purified proteins. To this end, we assembled a mammalian expression vector (referred to as P19-Tbx1-PA) coding for a fusion protein consisting of Tbx1 fused to protein A (PA) via a tobacco etch virus (TEV) protease cutting site (Figure 1a). We then generated stably transfected P19Cl6 cell lines expressing the Tbx1-PA fusion protein as well as a control protein without Tbx1 (P19-PA, Figure 1b). We selected P19CL6 cells because they can differentiate into cardiomyocytes upon treatment with DMSO [17] and, during this process, they express endogenous *Tbx1*, most clearly after 4 days of treatment (Figure S1). Thus, we treated P19-Tbx1-PA and P19-PA cell lines with DMSO for 4 days, and then we obtained nuclear extracts, which we subjected to affinity purification using IgG resin, and proteolytic elution, using TEV protease, to recover Tbx1-interacting protein complexes. Eluates were separated by SDS-PAGE (Figure 1c) and processed for Western blotting analyses. We tested antibodies against several candidate interactors, among which anti phospho-Smad1/5/8, because of its relevance to cardiovascular development and because of previous evidence of interaction with other T-box proteins [18], [19]. This antibody was positive when tested against the affinity-purified material (Figure 2a). Reciprocal coimmunoprecipitation of the two proteins transiently expressed in NIH 3T3 cells confirmed the interaction in mammalian cells (Figure 2b). We then extracted proteins from E9.5 wild type (WT) embryos and carried out co-immunoprecipitation with an antibody against Tbx1. Western blot analysis after immunoprecipitation revealed Smad1-specific immunoreactivity in co-immunoprecipitated material (Figure 2c). The interaction could not be demonstrated in cytosol extracts, indicating that it occurs in the nucleus (Figure 2d). We next tested whether mutant isoforms previously associated with a DiGeorge syndrome phenotype are capable of binding Smad1. We found that the mutant TBX1^F148Y^ (missense mutation in the T-box region [4]) can still bind Smad1, while the mutant TBX1^G310S^ (missense mutation in a conserved region downstream to the T-box region [4]) cannot (Figure 2e). In addition, we tested a T-box mutant (TBX1^G145R^), which has been shown to prevent DNA binding [20]. Also this isoform interacted with Smad1 (Figure 2e). Overall, these data suggest that the critical region for this interaction resides downstream to and outside the T-box region. We next tested whether Tbx1 could co-immunoprecipitated with other Smad proteins. We found that P-Smad2, Smad4, Smad5, and Smad6 do not interact with Tbx1 (Figure S2).

RETRACTED

**Figure 1:** Identification of Tbx1 interactors using affinity purification. Mouse P19-Cl6 embryonic carcinoma cells were stably transfected with plasmid expressing TEV-protein-A alone or C-terminally fused to Tbx1 and induced to differentiate with 1% DMSO. a) Constructs used to generate stably transfected P19CL6 cell clones. b) Western blot analysis of P19-Tbx1-PA and P19-PA (control) cell extracts. Proteins were separated by gel electrophoresis on 10% SDS-PAGE gel and immunoblotted with human IgG F(c), which recognize protein A. c) Colloidal coomassie-stained 10% SDS-PAGE gel containing nuclear extracts from P19-Tbx1-PA (lane 1) and P19-PA (lane 3) cells affinity purified by binding to IgG-Sepharose and then enzymatically eluted by cleavage with TEV protease. Compared with non-purified nuclear extract from Tbx1-TEV-PA cells (lane 2).

**Figure 2:** Tbx1 interacts with Smad1. a) Western blot analysis of affinity-purified nuclear extracts from P19-Tbx1-PA (lane 1) and P19-PA (lane 3) cells, compared non-purified nuclear extracts of P19-Tbx1-PA cells (lane 2), using an antibody anti-Phospho-SMAD1/5/8. b) Western blot analyses of reciprocal coimmunoprecipitation (IP) experiments using the antibodies indicated. NIH3T3 cells were co-transfected transiently with Tbx1-cmyc and Smad1-Flag expression vectors. c) Western blot analyses of nuclear extracts from wild type E9.5 mouse embryos immunoprecipitated with an anti-Tbx1 antibody (lanes 1 and 2) or with anti-rabbit IgG (lane 3) and revealed with an anti-SMAD1 antibody (lane 1 and 3) and an anti-Phospho-SMAD1/5/8 antibody (lane 2). d) Immunoblotting with anti-Smad1 antibody of nuclear extracts of wild type mouse embryos (E9.5) coimmunoprecipitated with anti-Tbx1 (NE-IP), total nuclear extracts (NE), total cytoplasmic extracts (CE), and cytoplasmic extracts coimminoprecipitated with anti-Tbx1 (CE-IP). e) Coimmunoprecipitation of WT TBX1, TBX1^G145R^, TBX1^F148Y^, TBX1^G310S^ and Flag-SMAD1 transiently transfected in NIH 3T3 cells. The TBX1^G145R^ and TBX1^F148Y^ mutants physically interact with Smad1, while TBX1^G310S^ is unable to bind Smad1 indicating that Glycine 310 is important for this interaction. f) Luciferase assay using Cos7 cells transfected with the SMAD-responsive reporter NTK-tetramer-luc. Transfected *SMAD1* activates the reporter while increasing amounts (5 to 100 ng) of co-transfected *TBX1* suppresses it.

RETRACTED

### Tbx1 modulates negatively the Bmp4- Smad1 signal transduction

To determine whether the interaction between Tbx1 and Smad1 has functional consequences, we overexpressed *Tbx1* and assessed the transactivation ability of Smad1. We carried out a luciferase assay in Cos-7 and C2C12 cells with the Smad-responsive reporter NTK-tetramer-luc, which contains four copies of a Smad consensus-binding element [21]. The reporter was activated by transfection of a *SMAD1* expression vector in Cos7 cells or by adding BMP4 to the culture media of C2C12 cells (Figure 2f and Figure S3, respectively). In both cases we observed that increasing amounts of transiently transfected *TBX1* is capable of suppressing Smad1- or BMP4-induced activation of the reporter (Figure 2f and Figure S3a). TBX1 expression did not affect the level of P-Smad1/5/8, Smad1 or the inhibitory Smad6 (Figure S4). To assess the role of transcriptional activity for the Bmp-Smad suppression activity, we expressed a mutant isoform of TBX1 (G145R) that carries a T-box mutation, which prevents DNA binding [20]. As shown in Fig. 3a, TBX1^G145R^ was unable to transactivate a T-box reporter, but it was still able to bind Smad1 (Figure 2e) and to suppress the Smad1 signaling in the luciferase assay, indicating that the anti-Smad activity of TBX1 is independent from transcriptional activity. We obtained the same results by activating the Smad reporter with BMP4 (Figure S3b).

**Figure 3:** Transactivation ability of Tbx1 is not required for Smad pathway suppression; Tbx1 interferes with Smad1/Smad4 binding. a) A luciferase assay showing the inability of the TBX1^G145R^ mutant to transactivate a T-box reporter construct in Jeg3 cells. Error bars indicate the standard error mean. b) A luciferase assay with a SMAD reporter showing that the mutant is capable of suppressing SMAD transactivation. c) Western blot analyses of nuclear extracts from C2C12 transfected with *Tbx1* and *SMAD1*-flag expression vectors (as indicated). The top two rows are samples immunoprecipitated with an anti-flag antibody. The bottom two rows are non-immunoprecipitated nuclear extracts from the same samples. Note the strong reduction of Smad4 co-immunoprecipitated with Smad1 in the presence of transfected TBX1.

RETRACTED

### Tbx1 interferes with Smad1-Smad4 binding

The Bmp-Smad1 signal transduction pathway requires binding of phosphorylated Smad1 to Smad4 to transactivate target genes [22]. To address the mechanism by which TBX1 suppresses Bmp-Smad signal transduction, we tested whether TBX1 interferes with SMAD1 to SMAD4 binding. To this end, we transfected *SMAD1* (tagged with *flag*) with or without increasing amounts of *TBX1* into BMP4-treated C2C12 cells and carried out co-immunoprecipitation of nuclear extracts using an anti-*flag* antibody. Western blot analysis of immunoprecipitated material using an anti-Smad4 antibody revealed, in the absence of transfected *TBX1*, the presence of Smad4, which was strongly reduced in samples co-transfected with *TBX1*. This effect was dosage-dependent (Figure 3c). In the same samples, the presence of TBX1 did not affect the level of Smad1, and did not affect the level of Smad4 in protein extracts before immunoprecipitation (Figure 3c). These data suggest that TBX1 inhibits the Bmp-Smad signaling pathway by interfering with Smad1-Smad4 interaction.

### Transgenic expression of Tbx1 in mice mimics the Bmpr1a loss of function phenotype

If TBX1 has an inhibitory effect on the Bmp-Smad1 pathway, then ectopic expression of *Tbx1* during mouse development may mimic loss of function phenotypes associated with loss of Bmp-Smad1 in the same tissues. To test the ability of Tbx1 to suppress Smad1 signaling during mouse development, we have used a mouse transgenic line, named COET (for Conditional OverExpression of *Tbx1*), expressing *Tbx1* upon Cre-mediated recombination [23]. We selected to cross this transgenic line with the *Ap2a^IREScre^*/+ driver [24] that expresses Cre in the ectoderm and neural crest tissues, both of which require Bmp-Smad1 signaling. Indeed, ectodermic deletion of the Bmp receptor gene *Bmpr1a* caused cleft lip [25], and conditional ablation of the same gene in neural crest cells caused cardiac outflow tract defects [26]. *Ap2a^IREScre^*/+; COET animals did not survive after birth (data not shown) and examination of E18.5 embryos revealed bilateral cleft lip (Figure 4a–a') and cardiac outflow tract (OFT) defects (Figure 4b–b') in all animals examined (n>20), and control animals exhibited a normal phenotype (Figure 4a and b, and data not shown). Moreover, consistent with the hypothesis of a suppression of the Bmp-Smad1 pathway, we observed reduced expression of the Bmp-Smad1 target gene *Msx1* [27] in E9.5 and E10.5 *Ap2a^IREScre^*/+;COET embryos (Figure 4c-f').

RETRACTED

**Figure 4:** Ectopic expression of Tbx1 in mouse embryos suppresses the Smad1 pathway in vivo. a–a') A *Ap2a^IRESCre^/+;Coet* embryo (a') at E18.5 shows bilateral cleft lip, compared with a control littermate (a). b–b') Three-dimensional reconstruction from digital images of histological sections of E16.5 hearts from control (b) and *Ap2a^IRESCre^/+;Coet* embryos. The cavities of the right (RV) and left (LV) ventricles, as well as the great arteries are shown in red. Note the large ventricular septal defect (VSD), and the common origine of the aorta and pulmonary arteries from the right ventricle, a condition known as double outlet right ventricle (DORV). (c–f') Whole-mount *in situ* hybridization analysis of *Msx1* expression in WT (c, d, e, f) and *Ap2a^IRESCre^/+;Coet* embryos (c', d', e', f') at E9.5 (c–d') and E10.5 (e–f'). Mutant embryos show reduced expression in the maxillary region (white arrows) and in the second pharyngeal arch (black arrows). (g) Cleft lip present in *Ap2a^IRESCre^/+;Coet* embryos (compare with panel a) is rescued by the *FSMAD1* transgene.

### Transgenic expression of Smad1 rescues partially the Tbx1 over expression phenotype

If the *Ap2a^IREScre^*/+;COET associated phenotype is due to functional depletion of Smad1, then providing an additional source of *Smad1* to the affected tissues may ameliorate the phenotype. To test this idea, we generated a mouse transgenic line that expresses *SMAD1* upon Cre-induced recombination (Figure S5). This transgenic line, named Fsmad1, was made with the same procedure and construct used to generate the COET line, except that we used a *SMAD1* cDNA instead of the *Tbx1* cDNA. *Ap2a^IREScre^*/+;Fsmad1 E18.5 embryos were grossly normal (data not shown), suggesting that additional *Smad1* expression in the ectoderm and neural crest, where endogenous *Smad1* is normally expressed, did not cause any obvious developmental anomaly. Next, we crossed COET;Fsmad1 mice with *Ap2a^IREScre^*/+ mice and examined the progeny at E18.5. No obvious abnormalities were detected in *Ap2a^IREScre^*/+;Fsmad1, but, as expected, all the *Ap2a^IREScre^*/+;COET examined (n = 7) exhibited cleft lip and cardiac outflow tract defects (similar to those shown in Figures 4a' and b', respectively). However, with one exception, none of the *Ap2a^IREScre^*/+;COET;Fsmad1 embryos examined exhibited cleft lip (n = 6, Figure 4g), however, they did exhibit outflow tract defects. Thus, excess *Smad1* expression was sufficient to rescue the cleft lip phenotype of *Ap2a^IREScre^*/+;COET embryos but not the heart phenotype.

RETRACTED

## Discussion

This study identified Smad1 as a novel interactor for the Tbx1 protein, and the only one that has been validated with endogenous proteins from embryos to date. Nowotschin et al. have shown that Tbx1 and Nkx2.5 interact in cell cultures, although they have not shown that the two endogenous proteins interact in embryo tissues [28]. While we did not map the regions of interaction between Tbx1 and Smad1, we demonstrate that a disease-associated missense mutation of Tbx1 in the C-terminal region of the protein is sufficient to prevent binding. These data suggest that perturbance of the Tbx1-Smad1 interaction may be part of the pathogenetic mechanism of DiGeorge syndrome.

Xbra, a Xenopus T-box protein, also binds to Smad1, and this interactions appears necessary to prevent Xbra from activating *Goosecoid*, but how exactly this is effected is unclear [18]. We show that Tbx1 modulates negatively Smad1-dependent transactivation by interfering with Smad1-Smad4 interaction. Using mouse transgenic models we could reproduce in vivo the Tbx1-mediated Smad1 repression. This could be revealed by the occurrence of a phenotype similar to that caused by loss of *Bmpr1a*, and by reduced expression of a BMP target, *Msx1*, in *Ap2a^IREScre^*/+;COET embryos. In these embryos, *Msx1* expression appeared downregulated only in some tissues. This may be due to tissue-specific Cre expression or to different, tissue specific mechanisms of *Msx1* regulation. In any case, the phenotype of ectopic expression of *Tbx1* could be partially rescued by transgenic expression of *Smad1* in the same tissues. The heart phenotype caused by ectopic expression of *Tbx1* in *Ap2a^IREScre^*/+;COET embryos could not be rescued by transgenic expression of Smad1. This could be because *Tbx1* ectopic expression in the neural crest may cause more perturbances than simply BMP suppression, perhaps in early development of neural crest cells destined to populate the heart.

Among the various developmental roles, Tbx1 is thought to maintain proliferation of mesodermally-derived cardiac progenitors of the second heart field (SHF) [14], a migratory cell population that enters the heart in a relatively late stage of its development [15]. Prall and coworkers [16] showed that *Smad1* ablation in the SHF enhances cell proliferation, and thus it has been proposed as a negative modulator of cardiac progenitors proliferation. Thus, it is conceivable, that Tbx1, by repressing Smad1, contributes to maintenance of cell proliferation. Recently it has been shown that Chordin (Chrd), a BMP antagonist, is a mild modifier of the *Tbx1* mutant phenotype. Indeed, Choi and Klingensmith [29] showed that loss of *Chrd* enhances the craniofacial phenotype of *Tbx1* mutants. This effect can be interpreted on the basis of our findings, i.e. at least part of the *Tbx1* mutant phenotype is due to excessive BMP signaling, thus removing an antagonist of BMP in a *Tbx1* mutant background further enhances the excess of BMP. The heart phenotype was not affected by *Chrd* mutation presumably because this gene is not expressed in heart tissues.

RETRACTED

Tbx1 has been shown to regulate, directly or indirectly, several of the major signaling systems, i.e. the fibroblast growth factor (FGF) signaling [7], [10], [30], [31], the Retinoic acid signaling [12], [31], the Delta-Notch1 signaling [32] and the BMP/Smad1 signaling (this work). Thus, we propose that Tbx1, by modulating positively the FGF and negatively the BMP-Smad1 signaling systems plays a central role in the homeostasis of cardiac progenitor cells of the SHF.

Finally, and perhaps most surprisingly, we show that the Smad1 modulatory effect of Tbx1 is not dependent upon DNA binding, therefore, this represents the first example of a transcription-independent function of a T-box transcription factor.

## Materials and Methods

### Constructs and cell lines

To generate the FSMAD1 transgene construct, the Flag-SMAD1 cDNA was excised from pCMV5-FlagSMAD1 [33] and cloned 3′ to a loxP-flanked neomycin resistance cassette with 3 polyadenylation-sites (the backbone plasmid is a kind gift from Drs. A. Simeone and F. Tuorto, Institute of Genetics and Biophysics, Naples). C2C12 cells were maintained in Dulbecco's modified Eagle's medium supplemented with 10% heat-inactivated fetal bovine serum. The human choriocarcinoma-derived placental JEG3 cell line was maintained in Minimum Essential Medium (SIGMA) supplemented with 10% fetal bovine serum. P19CL6 cells were grown in Dulbecco-Modified Minimal Essential Medium supplemented with 10% fetal bovine serum. For differentiation of P19CL6 cells, the culture medium was supplemented with 1% DMSO (Sigma-Aldrich). To generate stably transfected cell lines, 10^7^ P19CL6 cells were electroporated with 10 µg of DNA of an expression vector containing the cmv promoter driving a mouse Tbx1 cDNA fused with a TEV target site and a Protein A coding cDNA (the plasmid backbone has been described in ref. [34]. Using the same procedure but with an expression vector encoding the TEV site, Protein A but not Tbx1, we obtained a control cell line, P19-PA. Selection was performed using G418 (200 µg/ml). Resistant clones were picked, expanded and tested for expression of the transgenic proteins by western blotting.

RETRACTED

### Nuclear/Cytoplasmic Extract Isolation

Cells were cultured in 10 cm dishes until 60–70% confluence and transfected with Fugene6 (Roche) following the manufacturer protocol. After 24–48 h after transfection, cells were washed, scraped in cold PBS, and collected by centrifugation using a refrigerated centrifuge at 1000 rpm for 10 min. The pellet was resuspended in 5 pellet volumes of cold CE buffer (10 mM HEPES, 60 mM KCl, 1 mM EDTA, 0.075% v/v NP40, 1 mM DTT and 1X protease inhibitors, adjusted to pH 7.6), and centrifuged at 1400 rpm for 4 min. The nuclei were washed with 5 pellet volumes of cold CE buffer without detergent and spinned as above at 1400 rpm for 4 min. 2x pellet volume of NE buffer were added to the nuclear pellet incubating on ice for 30 min. Nuclear and cytosolic extracts were recovered spinning at maximum speed for 30 min to pellet any nuclei.

### Affinity purification

Native affinity purification was performed with strains P19-Tbx1-PA and P19-PA as previously described [35]. Nuclear extracts were transferred to Poly-Propylene Chromatography Columns (10 ml volume; Pierce), which contained 2 ml of pre-washed (with IPP150: 10 mM Tris-HCl, pH 8.0; 150 mM NaCl; 0.1% NP-40) IgG sepharose beads (Amersham). Columns were sealed and slowly rotated for 2 h at 4°C. After three washes with 10 ml of IPP150 buffer and one wash with 10 ml of TEV cleavage buffer (910 mM Tris-HCl, pH 8.0; 150 mM NaCl; 0.1% NP-40; 0.5 mM EDTA; 1 mM DTT), we added 1 ml TEV cleavage buffer and 10 µl of TEV enzyme (Amersham). Protein eluates were concentrated and loaded on a 10% SDS-acrylamide gel. Proteins were stained with colloidal coomassie or transferred into PVDF membrane (Amersham) for Western blotting analyses.

### Co-Immunoprecipitation

For co-immunoprecipitation experiments, cells were lysed at 4°C in Nonidet P-40 lysis buffer. Extracts were quantified using a modified Bradford procedure (Bio-Rad Laboratories, Hercules, CA). Co-immunoprecipitation of TBX1 and Flag-SMAD1 was accomplished using an antibody-coupling gel to precipitate the bait protein and co-immunoprecipitate the interacting prey protein. Anti-Tbx1 (Zymed Laboratories) or anti-Flag M2 antibody (SIGMA) was coupled to an amine-reactive gel (ProFound co-immunoprecipitation kit, Pierce) using slow agitation at 4°C O.N. The precipitated protein complexes were run on a 10% SDS-acrylamide gel, and analysed by Western blotting.

### Luciferase assay

Cos-7 cells were grown in 24-well plates and transfected with 100 ng of NTK-tetramer-luc vector [21], 100 ng of pCMV5-FlagSMAD1 and 5 ng to 100 ng of h-TBX1 (a TBX1 expression vector obtained by cloning a human cDNA into the CMV expression plasmid pCDNA3). C2C12 cells were grown in 24-well plates, transfected with 100 ng of NTK-tetramer-luc vector, 5 ng to 100 ng of h-TBX1 and stimulated with 50 ng/ml of Human recombinant BMP4. JEG3 cells were grown in 24-well plates and transfected using Fugene-6 (Roche) with 100 ng of 2xTtkGL2 vector [6], 5 ng of β-Gal-expression vector, and 100 ng of h-TBX1. In all the experiments, the total amount of transfected DNA was adjusted with empty vectors so that all samples received the same amount. Light emission of extracts was measured using a luminometer.

RETRACTED

### Mouse Mutants and Breedings

All the experiments involving mice were done according to a protocol reviewed and approved by the Institutional Animal Care and Use Committee of Institute of Biosciences and Technology, in compliance with the USA Public Health Service Policy on Humane Care and Use of Laboratory Animals.

The mutant AP2α^IREScre^ used in this study has been previously reported [36]. The COET transgenic mouse line has been described previously [23]. The FSMAD1 transgenic line was generated as follows. The FSMAD1 construct (described above) was linearized and electroporated into feeder-free E14Tg2A.4 embryonic stem cells (strain 129/Ola, BayGenomics). Cells were selected with G418, and 96 resistant clones were screened by southern blot using a probe specific for the Flag-SMAD1 sequence. 2 positive clones were tested for SMAD1 expression with Western blotting analysis after Cre recombination. One of the clones was injected into C57Bl6 blastocysts to obtain chimeric mice. Founders were backcrossed into the C57/Bl6 strain and maintained in a mixed genetic background C57/Bl6-129/Ola. FSMAD1 transgenic mice were crossed with COET mice (same genetic background) to generate COET; FSMAD1 mice for use in timed matings. COET; FSMAD1 mice were crossed with AP2α^IRESCre/+^ animals to generate embryos of the appropriate stage and genotype. The FSMAD1 transgene was genotyped with the following primers: 1) 5′- caaagacgacgatgacaagg -3′ and 2) 5′- agctcaaggccttttccagt -3′. Phenotypic analyses of mutant embryos were carried out by gross morphological analyses, embryo dissection and hystological analyses. In some cases, we used digital images of 10 mm-thick histological sections to carry out three-dimensional reconstructions using the software AMIRA 4.1.2 (Mercury Computer Systems).

### In-situ hybridization

Whole mount in situ hybridization was performed by standard methods. The mouse *Msx1* probe was kindly provided by James F. Martin (Institute of Biosciences and Technology, Houston).

RETRACTED

### Sources of antibodies and proteins

The anti-Tbx1 antibody was obtained from Zymed Laboratories; the anti-P-Smad1 (Ser463/Ser465) from Chemicon; The anti Smad1, P-Smad2 (Ser465/Ser467), Smad4, Smad5, and Smad6 where all purchased from Cell Signaling. Recombinant proteins BMP4 and TGFβ1 were obtained from R&D Systems.

## Supporting Information

Figure S1 Endogenous Tbx1 expression during cardiomyocite differentiation of P19Cl6 cells. RT-PCR analyses for the indicated mRNAs were performed on differentiating P19Cl6 cells. The Tbx1 amplification signal is more clearly evident starting from day 4 of differentiation.
(1.71 MB TIF)

Figure S2 P-Smad2, Smad4, 5, and 6 do not interact with Tbx1. Nuclear extracts of mouse P19-Cl6 cells induced to differentiate with 1% DMSO were purified by binding to IgG-Sepharose, digested with TEV protease and immunoblotted with (a) anti-Smad5, (b) anti-Smad4 and (c) anti-Smad6 antibodies. Lane 1: Purified nuclear extracts of cells expressing Tbx1-TEV-PA. Lane 2: Total nuclear extracts of cells expressing Tbx1-TEV-PA. Lane 3: Purified nuclear extracts of cells expressing TEV-PA alone. (d) NIH-3T3 cells were transiently transfected with TBX1, stimulated with 5 ng/ml of TGFβ1 for 1 hour and protein extracts were coimmunoprecipitated with anti-Tbx1 and immunoblotted with anti-Phospho-Smad2 antibody.
(8.51 MB TIF)

Figure S3 TBX1 or TBX1G415R are both capable of suppressing a Smad reporter after BMP4 activation. a) Luciferase assay using a Smad reporter (NTK-tetramer-luc) with C2C12 cells exposed to BMP4. Increased amounts of TBX1 expression vector DNA (from 5 ng to 100 ng) is associated with reduced luciferase activity. b) In a similar experiment, a vector encoding the mutant TBX1G145R isoform, which cannot transactivate a T-box reporter, has a similar capacity to suppress the Smad-reporter activity as the wild type isoform. The mean data are representative of three replicates for each condition and the error bars show the standard error.
(8.81 MB TIF)

Figure S4 TBX1 does not affect the level of P-Smad1/5/8, Smad1 and inhibitory Smad6. Western blot analyses of protein extracts from BMP4-induced and non induced C2C12 cells, with or without TBX1 transfection. None of the immunoreactivities tested in this figure is affected by TBX1 expression.
(7.23 MB TIF)

Figure S5 Generation of the FSMAD1 transgenic line. a) Schematic representation of the transgenic construct, which includes a chicken b-actin promoter, a loxP-flanked promoterless neo resistance cassette with 3 copies of a polyadenilation signal, and a cDNA encoding human SMAD1 tagged at the N-terminal with flag. b) Southern-blot of BamHI-digested DNA from ES-cell clones (parental and transgenic) probed with a Flag-SMAD1-specific probe. The position of the BamHI restriction sites is indicated on panel a. c) Western-blot analysis of protein extracts from parental and transgenic ES clones after transient Cre recombinase expression, using an anti-Flag antibody. A transgenic protein of the appropriate size is clearly evident in the transgenic cell line. d) PCR analysis of DNA from transgenic embryos using FSMAD1-specific the oligonucleotides 1) 5′- caaagacgacgatgacaagg -3′ and 2) 5′- agctcaaggccttttccagt -3′(the position of primers is schematically indicated on panel a.
(4.93 MB TIF)
